# A Linear Regression Prediction Model of Infectious Disease Spread Based on Baidu Migration and Effective Distance

**DOI:** 10.1155/2022/9554057

**Published:** 2022-06-14

**Authors:** Tianqi Zhou

**Affiliations:** School of Medical Devices, Zhejiang Pharmaceutical University, Ningbo, Zhejiang 315500, China

## Abstract

**Objective:**

To analyze the relationship between effective distance and epidemic spread trajectory and between arrival time and scale based on the COVID-19 data outbreak in Wuhan and thus to improve the prediction ability of the spread of infectious disease.

**Methods:**

Up to January 28, 2020, the reporting date, the onset date, and the cumulative number of confirmed cases of COVID-19 in each province and city were collected. Baidu migration data was used to calculate the effective distance from Wuhan city to other regions. The reporting date and onset date of the first diagnosed patient were taken as the arrival time, respectively, to establish a linear regression model of effective distance and arrival time. In different provinces and cities, the logarithm of the cumulative number of confirmed cases with a base of 5 was taken as the criteria to determine the level of the cumulative confirmed cases. Based on this, the linear regression model of effective distance and the level of cumulative confirmed cases in the provincial and municipal units was established.

**Results:**

The linear correlation between the reporting date of the first confirmed patient and the effective distance was not strong. The coefficients of determination (*R*^2^) for cities with and without the cities of Hubei Province were 0.36 and 0.44, respectively. And the linear correlation between the onset date of the first confirmed patient and the effective distance was strong. And the coefficients of determination (*R*^2^) for cities with and without the cities of Hubei Province were 0.67 and 0.83, respectively. And the linear correlation between the level of cumulative confirmed cases in the provincial and municipal units and the effective distance was strong, with an *R*^2^ of 0.87 and 0.84, respectively. The regression coefficients of each linear model were statistically significant (*P* < 0.001).

**Conclusion:**

The effective distance has a good fit with the model of the onset date of the first confirmed patient and the level of cumulative confirmed cases, which can predict the trajectory, time, and transmission range of the epidemic. It can be taken as the reference for the early warning, prevention, and control of sudden acute infectious diseases from a macro perspective.

## 1. Introduction

At present, there is no effective prediction method for the spread of sudden acute infectious diseases at home and abroad. And the related research mainly focuses on etiological and epidemiological factors. However, these factors are complicated. They are closely related to various factors, such as personal physical conditions, environment, and climate, which makes the epidemic difficult to grasp. And it is impossible to conduct early warning, effective prevention, and control [1]. Brockmann and Helbing proposed an effective distance model in 2013 [1, 2], which calculated the effective distance between regions through the passenger flow matrix of the air transportation network. The effective distance can not only contribute to determining the source of the outbreak of infectious disease but also significantly improve the ability to predict the transmission trajectory, arrival time, and transmission range of infectious diseases.

Due to the diversification of transportation in China, only air passenger flow cannot represent the whole movement of the population between different cities of China [3–6]. Therefore, instead of the air passenger flow used in the original model, Baidu migration data based on Location-Based Service (LBS), which provides accurate population flow data between provinces and cities [7–10], was selected and applied in this study to calculate the effective distance. And data on the COVID-19 outbreak in Wuhan as the outbreak site in December 2019 was collected. Linear regression models were established between effective distance and outbreak arrival time and between effective distance and transmission scale (cumulative number of the confirmed cases, which is represented by the level of the cumulative confirmed cases).

In this study, the effective distance calculated from Baidu migration data was used instead of the traditional geographical distance. Based on the effective distance from the outbreak site to different destinations, the effective distance was used to predict the trajectory, arrival time, and scale of epidemic spread when the epidemiological parameters of the epidemic were unknown. Moreover, it also provides a reference for future work in making early warning, prevention, and control of related epidemics.

## 2. Materials and Methods

### 2.1. Materials

The epidemic data was collected before January 28, 2020. The main data sources are as follows:

1. Public data from the official channels of the National Health Commission, provincial and municipal health commissions, and provincial, municipal, and district governments
2. Epidemic data compiled by The Paper (https://www.thepaper.cn/list_25635)
3. Epidemic data compiled by the “nCoV Epidemic Map” team (https://github.com/2020-nCoV/)
4. Baidu migration data

Record and gather data such as the cumulative number of confirmed cases of COVID-19, the date of reporting the first confirmed patient, the date of onset, and other related data in all provinces and cities. Instead of the air passenger flow, the population migration data provided by the Baidu migration platform, which could accurately represent the population flow among domestic cities, was used in the effective distance model. From December 1, 2019, to January 23, 2020, data on the proportion of emigration from Wuhan to 31 provinces (excluding Hong Kong, Macao, and Taiwan) and other cities across the country (the percentage of the population migration from Wuhan to a certain place in the total population flow of Wuhan) have been collected from the Baidu migration platform [1].

### 2.2. Methods

The effective distance from Wuhan to other cities was calculated by the effective distance model based on Baidu migration data, instead of the air passenger flow. In 2013, Dirk Brockmann and Dirk Helbing published the paper “The Hidden Geometry of Complex, Network-Driven Contagion Phenomena” in *Science*, exploring the relationship between air passenger flow and the crossregional spread of infectious diseases. In the study, the traditional geographic distance was replaced by the probability-oriented effective distance, which simplified the complex spatiotemporal pattern of infectious disease propagation with simple uniform wave propagation pattern, so that the trend of infectious disease spread could be accurately predicted even when the epidemiological characteristics were unknown. The validity and practicability of the model were verified through the data of influenza A (H1N1) in 2009 and SARS in 2003 [11]. The main calculation principles of the effective distance were as follows:

1. The crossregional transmission network of infectious diseases was represented by the air passenger flow matrix **P**, and *P*_*mn*_ represented the probability of outflow population from the node *n* to node *m*. That is, the percentage of population migration from node *n* to node *m*, which was calculated by dividing *X*_*mn*_ (the outflow population from *n* to *m*) by *X*_*n*_(the total outflow population from *n*). The calculation formula was

(1) $$\begin{array}{c} P_{mn}=\frac{X_{mn}}{X_{n}},\\ \sum P_{mn}=1,\;0\leq P_{mn}\leq 1 \end{array}$$

(2) The calculation formula of direct effective distance (*d*_*mn*_) from *n* to *m* was

(2) $$\begin{array}{c} d_{mn}=1-\text{lg}P_{mn}\geq 1 \end{array}$$

due to the asymmetry of population migration between regions, *P*_*mn*_ ≠ *P*_*nm*_ and *d*_*mn*_ ≠ *d*_*nm*_

(3) An ordered path from node *m* to node *n* was denoted as Γ = {*n*_1_, *n*_2,_⋯, *n*_*L*_}. The direct effective distance of the ordered path *λ*(Γ) was the sum of the effective distance of the ordered path. The calculation formula was

(3) $$\begin{array}{c} \lambda \left(\Gamma \right)=L-\text{lg}W\left(\Gamma \right) \end{array}$$

where *W*(Γ) = *P*_*n*_*L*_*n*_*L*−1__ × ⋯×*P*_*n*_2_*n*_1__ = ∏_*i*=1_^*L*−1^*P*_*n*_*i*+*j*_*n*_*i*__

(4) In the propagation network, the effective distance from any node *n* to node *m* was denoted as *D*_*mn*_. The calculation formula was as follows:

(4) $$\begin{array}{c} D_{mn}=\underset{\Gamma }{\min}\lambda \left(\Gamma \right),\\ D_{mn}\neq D_{nm} \end{array}$$

The effective distance was asymmetric, which reflected that random infectious diseases were more likely to spread to high-connected nodes and vice versa.

### 2.3. Statistical Analysis

Software, including Python3.8.3 and MySQL3.8.3, was used to capture and organize the data. The report date and onset date of the first confirmed COVID-19 patient were taken as the time when the disease appeared. Since the cumulative number of confirmed cases of COVID-19 varies greatly between different provinces and cities, for better data fitting, the logarithm of the cumulative number of confirmed cases (*N*) was taken as the base 5 and was defined as the level of the cumulative confirmed case (*M*), The calculation formula was as follows:

(5) $$\begin{array}{c} M=\text{lo}{\text{g}}_{5}N. \end{array}$$

SPSS 25.0 was used to establish the effective distance model and linear regression model to analyze the linear relationship between the effective distance and the arrival time of COVID-19, as well as the relationship between the effective distance and the level of cumulative confirmed cases of COVID-19.

## 3. Result

### 3.1. Effective Distance from Wuhan to Other Cities

From December 1, 2019, to January 23, 2020, the top three cities in terms of the proportion of the population moving out of Wuhan were as follows: Huanggang (12.61% of the population moving out), and Xiaogan (12.55%), Jingzhou (5.84%). The top three provinces in terms of the proportion of the population moving out of Wuhan were Hubei Province (62.62% of the population moving out), Guangdong Province (5.28%), and Henan Province (4.22%). In the effective distance model, the proportion of population movement from Wuhan to other provinces and cities was the probability of population mobility between two regions (*P*_*mn*_), from which the effective distance from Wuhan to each province and city could be calculated. Sorting the effective distances from the smallest to the largest, the effective distances of the top 5 cities are shown in Table 1.

### 3.2. Relationship between Effective Distance and Arrival Time

#### 3.2.1. Relationship between the Reporting Date of the First Confirmed Patient and the Effective Distance

The report date of the first confirmed COVID-19 patient in the city was taken as the arrival time of the COVID-19 outbreak in that place. The relationship between the effective distance from Wuhan to other cities and the arrival time of the epidemic is shown in Figure 1, and a linear regression analysis was performed on it. The data were fitted for the cities in Hubei Province and the cities outside Hubei Province, respectively. The regression equations were *T*_a_ = 0.42D + 11.07 and *T*_a_ = 0.71D + 7.84. As could be seen from Figure 1, the effective distance of some cities in Hubei Province, such as Huanggang and Jingzhou, was closer than that in Guangdong and Shanghai. However, the reporting date of the first patient was much later, which indicates that the reporting date of the first patient in some cities in Hubei Province was later than the actual arrival time of the disease. Excluding these cities in Hubei Province, the regression coefficient increased from 0.42 to 0.71, and the coefficient of determination *R*^2^ increased from 0.36 to 0.44. But the correlation was still not strong. The arrival of the disease in different cities was earlier than the reporting date of the first patient, especially in the cities of Hubei Province, the deviation of which was greater.

#### 3.2.2. Relationship between the Onset Date of the First Confirmed Patient and the Effective Distance

The onset date of the first confirmed patient in the city was used to determine the arrival time of the epidemic. If the onset date was missing, the reporting date of the first patient was recorded. The fitting situation of the onset date of the first confirmed patient and the effective distance is shown in Figure 2. Data fitting was performed for two cases, including the cities of Hubei Province and excluding the cities of Hubei Province. The regression equation of the fitted line including cities of Hubei Province was *T*_a_ = 1.31*D* + 32.37, and the coefficient of determination *R*^2^ = 0.67. The regression equation of the fitted line excluding cities of Hubei Province was *T*_a_ = 17.36*D* − 100.34 (reverse *x*- and *y*-axis fitting), and the coefficient of determination *R*^2^ = 0.83. The effect of the regression model excluding the cities of Hubei province was better, and the effective distance could explain the 83% variation of the model. When excluding the cities of Hubei Province and taking the onset date of the first confirmed patient as the arrival time of the epidemic, the degree of linear correlation between the effective distance and the arrival time was consistent with that in the effective distance model paper.

### 3.3. The Relationship between the Effective Distance and the Level of Cumulative Confirmed Cases

#### 3.3.1. Relationship between the Effective Distance and the Level of the Cumulative Confirmed Cases in the Provincial Units

From Figure 3, it could be found that there was a linear trend between the effective distance and the level of the cumulative confirmed cases in the provincial units. And linear regression analysis has been conducted. The results showed that the regression coefficient was -0.42 (95% *CI*:−0.44~−0.35). After the *t-*test, *t* = −16.64, *P* < 0.001, and regression equation: *M* = 5.12 − 0.42*D*. The coefficient of determination *R*^2^ was 0.87. *R*^2^ was 0.87, and the effective distance could respond to the 87% variation of the model. The effect of the regression model was relatively good.

#### 3.3.2. Relationship between the Effective Distance and the Level of the Cumulative Confirmed Cases in the Municipal Units

As shown in Figure 4, with the same method, a linear regression model was established to show the relationship between the effective distance and the level of the cumulative confirmed cases in the municipal units. The results were as follows: the regression coefficient was -0.37 (95% *CI*:−0.41~−0.35). After the *t*-test, *t* = −23.42, *P* < 0.001. The regression equation was *M* = 4.67 − 0.37*D*; the coefficient of determination *R*^2^ was 0.84. The effective distance could respond to the 84% variation of the model, and the effect of the regression model was relatively good. There was an obvious linear relationship between the effective distance and the level of cumulative confirmed cases in provinces and cities. The effective distance could explain most of the variation in the level of the confirmed cases and could be used to predict the scale of the epidemic spread.

#### 3.3.3. Relationship between the Effective Distance and the Level of the Cumulative Confirmed Case Levels of Each Province and City in Different Periods

As shown in Table 2, linear regression models were established between the level of cumulative confirmed cases in different periods of the outbreak of COVID-19 and the effective distance from Wuhan to other provinces and cities. And the stability and applicability of the relationship between the effective distance and the level of cumulative confirmed cases were further verified. The results showed that the regression coefficients of each model were statistically significant (*P* < 0.001). And from Table 2, the coefficients of determination of the models were high in all periods, except for that of municipal destinations on January 24 (*R*^2^ of 0.31), which was zero for confirmed cases in some cities due to early detection capacity or speed limitation. Therefore, it can be found that the method has good stability.

## 4. Discussion

At present, there are few studies on the warning, prevention, and control of sudden acute infectious diseases from the macroscopic perspective in China. Most of the existing research focuses on the pathogen, the patient, the infected population, and the close contact population. In the related research, the factors that influence the spread of the disease are very complex and difficult to grasp. They are closely related to the physical conditions of the virus carrier, the environmental conditions, the climate, and the physical conditions of the contact person [7–9]. However, if there are changes in the perspective of the research, the study on the spread of infectious diseases would be much clearer. From the macroscopic view, taking each city as a node, it will be possible to predict the spread of acute infectious diseases between cities [1].

From a macro perspective, this study takes population flow between cities as an entry point to explore the impact of population flow on the spread of sudden acute infectious diseases. The traditional geographic distance is replaced by the effective distance represented by population migration. The effective distance determines the process of crossregional spread of infectious diseases, which is unrelated to other parameters such as epidemiology and etiology. And a scientific basis is provided for making early warning, prevention, and control of sudden acute infectious diseases.

Baidu migration data is used in the effective distance model to analyze the COVID-19 outbreak data in Wuhan. The results show that, excluding the cities of Hubei Province and taking the onset date of the first confirmed patient as the arrival time, there is an obvious linear relationship between the effective distance and the arrival time. Meanwhile, there is also an obvious linear relationship between the effective distance and the level of cumulative confirmed cases in the provincial and municipal units. The model fitting degree is good, and the regression coefficients are all statistically significant (*P* < 0.001).

With the development of transportation diversity, the trajectory of an epidemic is not determined by the traditional geographical distance, according to the effective distance model. Instead, it is determined by the effective distance from the outbreak site to different destinations. Even if the epidemiological parameters of an epidemic are unknown, the effective distance can be used to predict the relative arrival time of the epidemic [4–8]. In this study, the linear relationship between the effective distance and the arrival time of COVID-19 has been demonstrated. It suggests that the macroscopic trajectory of the outbreak is generally based on the spread from the initial outbreak to its effective distance from near to far, which can provide guidance for outbreak prevention and control in the future. For example, after the confirmation of human-to-human transmission of COVID-19 on January 20, only the confirmed cases in Henan, Guangdong, and Zhejiang were reported on January 21. However, there were other cities in Hubei Province that had a closer effective distance. And it could be inferred that the epidemic had already appeared in some cities of Hubei Province theoretically, such as Huanggang and Xiaogan, whose effective distance was relatively short. Therefore, it is suggested that the investigation and prevention should be carried out as soon as possible, according to the effective distance of the prefecture-level cities.

According to the effective distance from Wuhan to other cities, the linear model of arrival time and effective distance can reflect the approximate transmission trajectory and the possible arrival time of the COVID-19 epidemic. And the number of possible infected cases in each city can be further predicted based on the linear model of cumulative confirmed cases, which provides guidance for the prevention and control of sudden outbreaks. As shown in Figure 1, the city extending on the right side has no reported case. According to the model, the report date of the first case in Yanbian, Jilin Province, is predicted to occur on January 25, 2020. And its official report time was January 29, 2020. Meanwhile, the first case in Aksu, Xinjiang, is predicted to occur on January 27, 2020. And its official report time was January 30, 2020.

Although the effective distance can explain the occurrence of most of the variations in the epidemic, it can only be used to estimate the arrival time roughly. With the analysis of the COVID-19 epidemic data, it can be found that the arrival time of the epidemic in the cities with the same effective distance may still be different. Due to the large differences in the incubation time of COVID-19 and the different prevention and control that have been conducted in different regions, the arrival time of the first confirmed patient varies greatly from region to region. The onset date recalled by the first confirmed patient is relatively subjective, which impacts the accuracy by taking it as the arrival time of the epidemic.

As shown in Figure 2, the effective distance from Shenzhen, Wenzhou, and Changsha to Wuhan is farther than some cities in Hubei Province. But the arrival time of the epidemic in these three cities is earlier. It indicates that there is a late reporting phenomenon in some cities of Hubei province, which is probably limited by the capacity and the speed of detection. And investigation and prevention should be carried out according to the effective distance between Wuhan and other cities.

Responding to most of the variation in the level of cumulative confirmed cases, the effective distance can be used for analyzing the scale of the epidemic and giving early warning. For example, in the official epidemic notification on January 23, 2020, confirmed cases have appeared in Beijing, Shanghai, Hunan, Guangdong, Jilin, Heilongjiang, etc. However, there was no confirmed case reported in the cities of Hubei Province, which has a closer effective distance, such as Xianning, Xiangyang, and Ezhou. In theory, the number of confirmed cases in these cities should be higher. And the investigation, prevention, and control should be strengthened in these areas. In addition, the reality is much more complicated with many exceptions. As shown in Figure 4, Wenzhou, which deviates far from the fitting line, has a farther effective distance to Wuhan than Beijing, Chongqing, and Shanghai. However, the cumulative number of confirmed cases in Wenzhou is comparable to these cities. Based on the analysis of the existing information, the reason for the phenomenon may be that the proportion of people doing business from Wuhan to Wenzhou is relatively high. During this period, there will be more social activities. And persons in Wenzhou are likely to have contact with a large group of people, which increases the probability of infection.

The limitations of the study are as follows: (1) there exist some limitations in Baidu migration data, such as the strong bias of the collected groups [1], which causes deviations in the calculation of the effective distance. (2) Reporting dates of the first confirmed patients in different cities are relatively concentrated, and the onset dates reported by the patients themselves are highly subjective, so there will be deviations taking the two factors as the arrival time of the epidemic. (3) Determination coefficient of arrival time and effective distance model is not very high, which indicates that the single variable of effective distance cannot explain the variation of the epidemic arrival time. In the future, more accurate data can be considered. Other parameters, such as transmission speed and relevant macroscopic quantities, can be used for modeling to improve the predictive ability of the spread of infectious diseases.

COVID-19 outbreak data demonstrate the practical use of effective distance models in predicting the spread of sudden acute infectious diseases. In the future, the model can be used in the repeated outbreaks of the epidemic that occurs in a certain region. With the latest crowd flow data, it is possible to predict the risk of outbreaks in different cities in the context of population movement. And the scientific basis for epidemic traffic control in every city is provided. Meanwhile, effective distance methods can also be used in other related communication phenomena, such as the proliferation of new technologies and the spread of cyberviolence and rumors, which is playing an increasingly important role in a society full of communication and connection.

## Figures and Tables

**Figure 1:** The relationship between the report date of the first patient and the effective distance.

**Figure 2:** The relationship between the date of onset of the first patient and the effective distance.

**Figure 3:** The relationship between the effective distance and the level of the cumulative confirmed cases in the provincial units.

**Figure 4:** The relationship between the effective distance and the level of the cumulative confirmed cases in the municipal units.

**Table 1:** Effective distance.

City	Effective distance
Huanggang	2.96548693124562
Xiaogan	3.04547821456361
Jingzhou	3.71547892146645
Xianning	3.84567841654426
Ezhou	4.12544458775589

**Table 2:** Linear regression model between the effective distance and the level of cumulative confirmed cases in different periods.

Destination	Data (month-day)	Regression coefficient (95% CI)	*t*-test	*P* value	Regression equation	*R* ^2^
Provincial level	01-24	-0.32 (-0.36~-0.25)	-11.37	0.000	*M* = 3.00 − 0.31*D*	0.81
	01-31	-0.36 (-0.40~-0.30)	-14.47	0.000	*M* = 4.11 − 0.35*D*	0.87
	02-07	-0.38 (-0.43~-0.33)	-15.84	0.000	*M* = 4.64 − 0.38*D*	0.89
	02-14	-0.42 (-0.46~-0.36)	-17.14	0.000	*M* = 4.93 − 0.41*D*	0.90
	02-21	-0.43 (-0.47~-0.37)	-16.78	0.000	*M* = 5.12 − 0.42*D*	0.91
Municipal level	01-24	-0.19 (-0.25~-0.12)	-5.67	0.000	*M* = 1.73 − 0.18*D*	0.31
	01-31	-0.33 (-0.36~-0.28)	-18.11	0.000	*M* = 3.62 − 0.32*D*	0.76
	02-07	-0.36 (-0.38~-0.32)	-20.23	0.000	*M* = 4.34 − 0.35*D*	0.80
	02-14	-0.38 (-0.41~-0.34)	-22.53	0.000	*M* = 4.64 − 0.37*D*	0.83
	02-21	-0.39 (-0.41~-0.35)	-23.55	0.000	*M* = 4.7 − 0.38*D*	0.84

## Data Availability

The data used to support the findings of this study are included within the article.
